The article "Evaluation of the Practical Effects of Environmental Measures in the Conservation of Architectural Heritage in Yan'an Based on Recurrent Neural Networks" was published in 2022. Journal: J Environ Public Health.

# Evaluation of the Practical Effects of Environmental Measures in the Conservation of Architectural Heritage in Yan'an Based on Recurrent Neural Networks

**DOI:** 10.1155/2022/3749482

**Published:** 2022-09-12

**Authors:** Li Wang

**Affiliations:** School of Art and Media, Xi'an Technological University, Xi'an, Shaanxi 710032, China

## Abstract

Yan'an is one of the “two holy places” of the Chinese nation and the Chinese revolution and is one of the first cities of historical and cultural significance and an outstanding tourist city in China, as announced by the state council. The evaluation of the effectiveness of environmental conservation is one of the very important elements of the conservation of Yan'an's architectural heritage. However, the existing evaluation methods cannot provide new solutions for decision-making, the meaning of the comprehensive evaluation function is unclear, the naming clarity is low, there is less quantitative data and more qualitative components, and the results are not easily convincing. This paper proposes a method for evaluating the practical effects of environmental class measures in the conservation of Yan'an's architectural heritage based on recurrent neural networks. The recurrent neural network makes full use of the memory function in the network, considers the causal relationship of the actual effect, and efficiently evaluates the existing measures. In comparison with factor analysis and hierarchical analysis, this paper has greater applicability in evaluating the practical effects of environmental measures in the conservation of Yan'an's architectural heritage and is basically consistent with the results of the theoretical analysis. It provides a scientific basis for the construction and implementation of environmental measures for the architectural heritage of Yan'an.

## 1. Introduction

Architectural cultural heritage is the artifacts and monuments that humanity has conserved during historical development. It is an important part of humanity's historical and cultural heritage. In recent years, with the increasing importance attached by the state to the protection of cultural heritage, the state's financial resources for cultural heritage protection have been increasing year by year, so that various types of cultural relics, especially national and provincial cultural heritage protection units, have been effectively protected, which has strongly promoted the development of cultural heritage protection [1]. However, due to factors such as urban economic development and environmental changes, the current situation of cultural heritage protection units in China is still worrying, with some of them in serious disrepair and some on the verge of destruction, causing great difficulties for the protection of cultural heritage at the grassroot level, and to a certain extent affecting the development of urban cultural construction and the development of cultural heritage protection. The establishment of an effective evaluation system in terms of urban heritage conservation can help cities determine the future direction of development and better develop their economies, while avoiding conflicts with cultural heritage conservation work [2, 3]. The government and all facets of society have worked extremely hard in recent years to implement environmental measures for the rescue and conservation of Yan'an's architectural heritage. They have also taken numerous beneficial and efficient conservation measures to strengthen and improve this important work, which has now entered a comprehensive and holistic stage of conservation and has yielded many significant accomplishments and invaluable experiences.

While more and more attention is being paid to the conservation and heritage of Yan'an's architectural and cultural heritage, the conservation and use of revolutionary heritage is somewhat lacking, and special research into the conservation of this heritage is weak. Yan'an is also one of the three major educational bases for patriotism, revolutionary tradition, and the spirit of Yan'an and has the largest number, largest scale, longest span, highest level, and richest content of revolutionary heritage groups in the country. The architectural heritage addresses of Yan'an are the physical witness to the glorious revolutionary history of Yan'an and the material carrier of the Yan'an spirit [4]. Among the revolutionary base cities of the country, Yan'an has the largest, most numerous, most complete, and richest heritage preserved, with supremacy, uniqueness, and uniqueness [5]. However, due to the destruction of the war years, the negligence in the protection of architectural and cultural heritage in the special historical stage after the founding of the country, the damage caused by natural disasters, the preservation condition, and the preservation environment of some heritage need to be improved. The preservation of the architectural heritage of Yan'an is of great importance in remembering the past, educating the present, and reviving the future [6].

The conservation of Yan'an's architectural heritage today is inevitably impacted by urbanization, economic development, tourism promotion, and other aspects, making its preservation status and the development of environmental work in architectural heritage conservation serious challenges [7]. In the context of China's rapid urbanization, the revolutionary heritage of the Yan'an architectural heritage is also facing conservation and management problems such as natural aggression, deterioration, and environmental pollution, especially as the large-scale urban construction in Yan'an in recent years has posed a very serious threat to the preservation of the revolutionary heritage and its environment [8, 9]. Therefore, the conservation and research of the architectural heritage of Yan'an cannot be delayed. Moreover, from the perspective of cultural heritage and humanity, the conservation research of the architectural heritage of Yan'an also has certain theoretical and practical significance for the conservation and sustainable development of the revolutionary heritage. In addition, with the rise in economic power, residents are demanding a renewal of their living environment [10]. However, the socioeconomic costs of relocating residents within the heritage area are increasing, and as relocation is not possible, residents are forced to seek self-renewal in their neighborhood. However, as the heritage is only bounded by the conservation area, but not by the surrounding area, individual residents' spontaneous construction behavior is bound to destroy the landscape of the heritage area. To protect it from the threat posed by the city's rapid development, it is vital to take into account the general planning of the Yan'an architectural legacy at this time [11, 12]. The evaluation of the protection effect of Yan'an architectural cultural heritage should be based on environmental protection, and the method of comparative analysis, factor analysis, and hierarchical analysis should be adopted to comprehensively analyze the effectiveness of the evaluation measures.

The development and implementation of policies related to the implementation of environmental measures in the architectural heritage of Yan'an directly affects the heritage and development of the architectural heritage of Yan'an and plays a decisive role in the effectiveness of the conservation of the architectural heritage of Yan'an [13]. The evaluation of policy effects is in turn one of the key steps towards policy optimization and continuous improvement of policy capacity. Based on factor analysis and hierarchical analysis, a dynamic evaluation of the effectiveness of conservation of Yan'an's architectural heritage can provide a direct basis for evaluating the science and effectiveness of environmental measures in Yan'an's architectural heritage by vertically exploring the changes in the survival of Yan'an's architectural heritage and horizontally comparing the differences in the implementation of environmental measures in different regions of Yan'an's architectural heritage to explore the causes and policy differences [14, 15]. However, the existing evaluation methods do not provide new solutions for decision-making, the meaning of the comprehensive evaluation function is unclear, naming clarity is low, quantitative data is scarce, qualitative components are numerous, and the results are not easily convincing. Starting from the connotation of holistic conservation, it has become a new academic proposition and proposition of the times to scientifically evaluate the effect of the conservation of Yan'an architectural and cultural heritage and to improve the policy level, policy capacity, and conservation performance of the conservation of Yan'an architectural and cultural heritage [16, 17]. The analysis of Yan'an's architectural heritage's conservation effects can advance cultural heritage theory, serve as a foundation for the scientific preservation of architectural heritage, and improve architectural heritage direction prediction. This paper proposes a method for evaluating the actual effects of environmental-type measures in the conservation of Yan'an's architectural heritage based on recurrent neural network (RNN). In comparison with factor analysis and hierarchical analysis, the method is more applicable to the evaluation of the practical effects of environmental measures in the conservation of architectural heritage in Yan'an and is basically consistent with the results of the theoretical analysis. It provides a scientific basis for the construction and implementation of environmental measures for the architectural heritage of Yan'an.

## 2. Related Works

The process of conserving architectural history involves a variety of diverse substrates, highly heterogeneous sets of elements, and several distinct conservation circumstances. Due to general resource shortages and the distinctive qualities of cultural heritage assets, its sustainability has recently become a pertinent concern. Gulotta and Toniolo [18] use the creation of the test site as an appropriate example of a complex surface in their report on the design of a conservation project for the Renaissance façade of the Monza Cathedral. With the goal of identifying the most significant stakeholders and educating them about their critical role in the management of built heritage, Wang et al. [19] selected a tourist-built heritage as a study topic. The study's findings indicated that key players in the development of the built heritage of tourism's sustainability included local government, the federal government, real estate development companies, professional groups, architectural heritage conservation management, and architectural heritage construction companies. Lidelöw et al. [1] categorized and assessed the discovered research in light of two crucial components of such investigations: energy analysis and cultural heritage value analysis. The results highlight the importance of properly articulating and comparing cultural heritage values to accepted conservation principles or practices when thinking about energy improvements.

When developing solutions to reconcile the need to improve energy production using renewable energy with the requirement to conserve the built history and landscape, the designer should be guided by the features of each structure and its setting. A preliminary analysis of the restoration project can increase the building's sustainability and stop any irreparable alterations to the cultural property. De Medici [20] established evaluation standards for the installation of solar systems in preindustrial buildings using the Italian case study and recommendations for enhancing the sustainability of energy generation. Aigwi et al. [21] analyzed the distribution of significant government funding sources for their conservation, as well as the implications of this distribution for future architectural heritage conservation in provincial areas of New Zealand. They evaluate the dispersion of New Zealand's historic structures as well. In order to create sustainable societies, Salameh et al. [22] looked into and emphasized the intrinsic significance of heritage preservation from an environmental, economic, and social standpoint. From an architectural and urban standpoint, the study assesses a unique instance of historical preservation in the Palestinian city of Nablus.

## 3. Models and Evaluation Methods

### 3.1. RNN Neural Network Introduction

Traditional machine learning algorithms mainly rely on manually collected features, while fully connected neural network-based approaches have too many parameters and cannot take advantage of time series data in the data. The ability of RNN to access time series information in data and to express semantic information in depth has been fully exploited as more efficient RNN structures have been proposed, leading to advancements in speech recognition, language modeling, machine translation, and time series analysis [23, 24]. A type of recursive neural network known as an RNN accepts sequence data as input, recurs in the direction of sequence evolution, and connects all of its nodes (also known as recurrent units) in a chain. RNN is more effective in learning nonlinear characteristics of sequences because they share parameters, are remembered, and are Turing complete. RNN is first used to describe the relationship between a sequence's current output and its past information [25, 26].

A recurrent neural network, in terms of network architecture, keeps track of prior data and applies that data to affect the output of subsequent nodes. In other words, a RNN's hidden layers are interconnected, and their inputs contain both the outputs of the input layers and the outputs of the hidden levels from earlier in time [27]. The RNN complex can be conceptualized as the outcome of endless replication of the same neural network structure. A RNN delivers an output for each moment of input paired with the current state of the model. RNN shares parameters at multiple temporal positions, similar to how convolutional neural networks do, allowing sequences of any length to be processed with a limited amount of parameters [28].

The development of RNN has significant effects on the training of models. After unfolding a sequence of length *N*, the RNN can be viewed as a feedforward neural network with *N* intermediate layers, as shown in Figure 1. Since there are no circular links in this feedforward neural network, it may be trained directly using a back propagation technique without the use of any additional optimization procedures. Backpropagation through time is the name of this training technique, which is most frequently used to train the RNN.

On the basis of the aforementioned model, the forward propagation algorithm for RNN is presented. For any sequence moment *t*, the hidden state *h*^*t*^ is obtained from *x*^*t*^ and *h*^*t*−1^:

(1) $$\begin{array}{c} h^{t}=\sigma \left(z^{\left(t\right)}\right)=\sigma \left({Ux}^{\left(t\right)}+{Wh}^{\left(t\right)}+b\right), \end{array}$$

where the bias term is *b* and is the RNN's activation function, generally tanh. The following is the expression for the model's output, *o*(*t*), at sequence moment *t*:

(2) $$\begin{array}{c} O^{t}={Vh}^{\left(t\right)}+c. \end{array}$$

The final output of our prediction at sequence moment *t* is:

(3) $$\begin{array}{c} {\overset{\wedge }{y}}^{\left(t\right)}=\sigma \left(o^{\left(t\right)}\right). \end{array}$$

Usually, since RNNs are classification models for recognition classes, this activation function above is typically softmax. By means of loss function *L*^(*t*)^, we can determine the loss of the model at the present time using loss functions, such as log-likelihood loss functions and cross-entropy loss functions.

The RNN backpropagation algorithm can be easily derived using the foundation of the RNN forward propagation technique. The appropriate RNN model parameters *U*, *W*, *V*, *b*, and *c* are obtained by iterating through one round of gradient descent. RNN backpropagation is also known as BPTT because we are backpropagating over time (backpropagation through time). Since we update the same parameters when backpropagating, this BPTT is obviously significantly different from the DNN in that all *U*, *W*, *V*, *b*, and *c* are shared across the sequence. The cross-entropy loss function is used as the loss function in this instance; the softmax function is used as the activation function for the output, and the tanh function is used as the activation function for the hidden layer [29, 30]. The final loss *L* for the RNN is as follows because there are loss functions at each location in the sequence:

(4) $$\begin{array}{c} L=\overset{\tau }{\underset{t=1}{\sum }}L^{\left(t\right)} \end{array}$$

where *τ* is the total time step of the sequence.

The gradient is next found for *V* and *c* and can be expressed as:

(5) $$\begin{array}{c} \frac{\partial L}{\partial c}=\overset{\tau }{\underset{t=1}{\sum }}\frac{\partial L^{\left(t\right)}}{\partial c}=\overset{\tau }{\underset{t=1}{\sum }}\frac{\partial L^{\left(t\right)}}{\partial o^{\left(t\right)}}\frac{\partial o^{\left(t\right)}}{\partial c}=\overset{\tau }{\underset{t=1}{\sum }}{\overset{\wedge }{y}}^{\left(t\right)}-y^{\left(t\right)} \end{array}$$

(6) $$\begin{array}{c} \frac{\partial L}{\partial V}=\overset{\tau }{\underset{t=1}{\sum }}\frac{\partial L^{\left(t\right)}}{\partial V}=\overset{\tau }{\underset{t=1}{\sum }}\frac{\partial L^{\left(t\right)}}{\partial o^{\left(t\right)}}\frac{\partial o^{\left(t\right)}}{\partial V}=\overset{\tau }{\underset{t=1}{\sum }}\left({\overset{\wedge }{y}}^{\left(t\right)}-y^{\left(t\right)}\right){\left(h^{\left(t\right)}\right)}^{T} \end{array}$$

However, the gradient calculation of *W*, *U*, and *b* is more complicated. The gradient loss during backpropagation at a sequence location *t* is influenced by both the gradient loss corresponding to the output at the present position and the gradient loss at the sequence index point *t* +1, as can be shown from the RNN model [31]. It is necessary to backpropagate the gradient loss for *W* at a sequence location *t* step by step. The gradient of the hidden state at sequence index point *t* is given as follows:

(7) $$\begin{array}{c} \delta^{\left(t\right)}=\frac{\partial L}{\partial h^{\left(t\right)}} \end{array}$$

(8) $$\begin{array}{c} \delta^{\left(t\right)}=\frac{\partial L}{\partial o^{\left(t\right)}}\frac{\partial o^{\left(t\right)}}{\partial h^{\left(t\right)}}+\frac{\partial L}{\partial h^{\left(t+1\right)}}\frac{\partial h^{\left(t+1\right)}}{\partial h^{\left(t\right)}}=V^{T}\left({\overset{\wedge }{y}}^{\left(t\right)}-y^{\left(t\right)}\right)+W^{T}\delta^{\left(t+1\right)}\mathrm{diag}\left(1-{\left(h^{\left(t+1\right)}\right)}^{2}\right) \end{array}$$

For *δ*^(*τ*)^, since it is not followed by any other sequence index, there is

(9) $$\begin{array}{c} \delta^{\left(\tau \right)}=\frac{\partial L}{\partial o^{\left(\tau \right)}}\frac{\partial o^{\left(\tau \right)}}{\partial h^{\left(t\right)}}=V^{T}\left({\overset{\wedge }{y}}^{\tau }-y^{\left(\tau \right)}\right) \end{array}$$

Thus, the expression for the gradient of *W*, *U*, and *b* is calculated as

(10) $$\begin{array}{c} \frac{\partial L}{\partial W}=\overset{\tau }{\underset{t=1}{\sum }}\frac{\partial L^{\left(t\right)}}{\partial h^{\left(t\right)}}\frac{\partial h^{\left(t\right)}}{\partial W}=\overset{\tau }{\underset{t=1}{\sum }}\mathrm{diag}\left(1-{\left(h^{\left(t\right)}\right)}^{2}\right)\delta^{\left(t\right)}{\left(h^{\left(t-1\right)}\right)}^{T} \end{array}$$

(11) $$\begin{array}{c} \frac{\partial L}{\partial U}=\overset{\tau }{\underset{t=1}{\sum }}\frac{\partial L^{\left(t\right)}}{\partial h^{\left(t\right)}}\frac{\partial h^{\left(t\right)}}{\partial U}=\overset{\tau }{\underset{t=1}{\sum }}\mathrm{diag}\left(1-{\left(h^{\left(t\right)}\right)}^{2}\right)\delta^{\left(t\right)}{\left(x^{\left(t\right)}\right)}^{T} \end{array}$$

(12) $$\begin{array}{c} \frac{\partial L}{\partial b}=\overset{\tau }{\underset{t=1}{\sum }}\frac{\partial L^{\left(t\right)}}{\partial h^{\left(t\right)}}\frac{\partial h^{\left(t\right)}}{\partial b}=\overset{\tau }{\underset{t=1}{\sum }}\mathrm{diag}\left(1-{\left(h^{\left(t\right)}\right)}^{2}\right)\delta^{\left(t\right)} \end{array}$$

Depending on the RNN model, the formula for natural forward-backward propagation will be somewhat different, but the principles are basically similar. In reality, if the sequence is too long, on the one hand, it will cause gradient dissipation and explosion during optimization; on the other hand, the unfolded feedforward neural network will take up too much memory. As a result, a maximum length is set, and when the length reaches that limit, the sequence is truncated.

### 3.2. Based on the Assessment Framework of Environmental Measures in Yan'an Architectural Heritage Protection Work

In China's urban redevelopment process, architectural heritage, particularly tourism legacy, has been destroyed due to a lack of stakeholder protection. Therefore, identifying significant stakeholders is urgently needed in order to fulfill the duty of conservation. Based on the requirements of environmental measures in the conservation of architectural heritage in Yan'an, the basic components of the comprehensive evaluation of the conservation of architectural heritage units in Yan'an are summarized into four factors: the current state of conservation of architectural heritage units in the urban area and the environmental conditions around them, the protection of the historic and cultural style neighborhoods, the protection and support of the unique style culture, and the remediation of urban safety hazards that threaten the conservation of cultural heritage. On this basis, the framework of the evaluation index system is established. In order to provide a simple decision-making method for complex decision-making problems with multiple objectives, multiple criteria, or unstructured characteristics, this deep learning method uses less quantitative information to mathematically represent the thinking process of decision-making based on an in-depth analysis of the nature of complex decision-making problems, the influencing factors, and their intrinsic relationships. It is especially appropriate in circumstances where it is challenging to measure a decision's outcome properly and directly. The important details of the evaluation process are analyzed below, and the overall evaluation details are shown in Figure 2.

Firstly, the content of the evaluation should be clear. The soundness, the reasonableness, and the clarity of the evaluation content directly determine the scientific and accurate results of the evaluation. The key to evaluating the effectiveness of the holistic conservation of Yan'an's architectural heritage is to understand the meaning of “holistic” and “conservation” and to focus on these two aspects. At the same time, the content of the evaluation should be as simple and clear as possible to minimize artificial ambiguity in the evaluation process, while ensuring that the content is sound and reasonable. If the government subsidizes and invests in the preservation of historic buildings, it will save the future preservation of historic buildings and help revitalize the local economy.

Secondly, the indicators are scientific and practical. The evaluation of effects, as a scientific process of evaluating conservation results, should have a scientific attitude and a comprehensive evaluation method. Effectiveness evaluation, as a means of enhancing the conservation performance of Yan'an's architectural heritage, should change in connotation accordingly with the different types of heritage and the needs of conservation. However, the unrealistic nature of an absolutely scientific and reasonable index system, in turn, determines the relativity in the process of constructing an index system for evaluating the effectiveness of the holistic conservation of Yan'an's architectural heritage. Therefore, the indicators should be based on relative scientific rationality and strengthen their practicality.

Finally, operability of any scientific and perfect indicator system must be tested by evaluation practice. When setting indicators, the practical operability of the selected indicators should be considered, and the selection of indicators should also take into full consideration the actual needs of research and the possibility of data and information collection. Indicators that have some value but are not operational, and those that may inconvenience assessment experts and create difficulties for subsequent research on the indicator system, should be avoided as far as possible in the selection process. It is important to use as few and simplified indicators as possible to reflect the overall conservation effect of Yan'an's architectural heritage and to ensure that the evaluation process is simple, easy to follow, and operational.

## 4. Discussion and Analysis of Results

With the increasing attention to the protection and inheritance of architectural and cultural heritage, the protection and utilization of revolutionary heritage is still insufficient, and the special research on this kind of heritage protection is still weak; especially, the actual effect evaluation of environmental measures in the protection of Yan'an architectural heritage is still weak. The architectural heritage of Yan'an should be protected with targeted conservation techniques, while daily maintenance and conservation of Yan'an buildings should be strengthened, and regular safety treatments should be applied to the heritage body and its protective structures. In the face of rapid urban development and construction, an overall plan must be drawn up for the area around the heritage; on the basis of the current urban master plan, a scientific and reasonable protection zone should be drawn up, and in addition to setting up a protection zone, a construction control zone should be defined on its periphery, and corresponding protection management regulations and measures should be strictly formulated.

Hierarchical analysis is a comprehensive evaluation method [32]. Its essence is a process of decomposing complex problems. The process combines the basic steps that humans take when making decisions, namely, decomposition, judgement, and synthesis. To a certain extent, it reduces the subjectivity of the decision maker. The five steps of hierarchical analysis are analyzing the relationship between the factors in the system and establishing a system hierarchy, creating a comparison matrix by comparing components at the same level two by two, figuring out the relative weights of the elements in the comparison matrix at each level, evaluating the consistency of the comparison matrix, and calculating the synthetic weights under the whole system and calculating the total score of the evaluated object. A line that represents the data's median runs through the center of a box-line diagram. The box-and-line diagram is first used to portray the evaluation of the actual effect of environmental-type measures in the conservation of Yan'an's architectural heritage. The boxes contain 50% of the data since the top and bottom of the boxes correspond to the top and lowest quartiles of the data, respectively. Therefore, the height of the box partially indicates how much the data fluctuate. The maximum and minimum values of the data set are then represented by the top and bottom edges. There are occasionally data points outside the box that can be viewed as “outliers.” Figure 3 depicts the box-line diagram used in the hierarchical analysis method, which uses statistics like the median, 25th and 75th percentiles, and upper and lower boundaries to describe the overall distribution of the data. It finds that too many outliers reduce the effectiveness of the evaluation. These statistics are used to create a box plot, with the majority of the normal data located inside the box and the aberrant data located outside the upper and bottom box limits. No matter what policies and measures are formulated, the ultimate purpose is to better realize the protection, inheritance, and development of architectural heritage. The key is whether these policies and methods are implemented, whether they are practical, and whether they achieve the desired goals.

Hierarchical analysis does not offer fresh options for making decisions. Less quantitative information and more qualitative elements are difficult to persuade. When there are numerous indications, the data statistics are huge and it is challenging to identify the weights [33]. A comparison of the simulation responses is shown in Figure 4, which shows that the difference between the evaluation effect and the true fitted value is too large.

The study of statistical methods that separate common components from collections of data is known as factor analysis. The discovery of hidden representative components among numerous variables is made possible by factor analysis. The number of variables can be decreased, and the relationship between the variables' hypotheses can be investigated by combining variables with similar characteristics into a single factor. The box-line plot of the factor analysis method is shown in Figure 5, where it can be observed that the data fluctuates considerably, which is not conducive to the evaluation of actual effects. For a large sample with a typical normal distribution, the median lies in the middle of the upper and lower quartiles, and the box plots are symmetrical around the median, providing more evidence of the skewness of the data. The distribution is increasingly skewed the farther the median is from the upper and lower quartile centers. A right-skewed distribution results from outliers concentrated on the side of larger values; a left-skewed distribution results from outliers concentrated on the side of smaller values.

When calculating factor scores, the least squares method is used, which can sometimes fail. When the sign of the factor loadings of the principal components has positive and negative signs, the meaning of the integrated evaluation function is unclear and the naming clarity is low [34]. A comparison of the simulation responses is shown in Figure 6, which shows that the evaluation effect differs too much from the true fitted value.

Finally, the RNN method was used to build an evaluation model for environmental-type measures in architectural heritage conservation work. Case line with the upper and bottom boundaries of the boxes representing the upper and lower quartiles of the data, respectively, and the boxes containing 50% of the data, Figure 7 compares the shapes of multiple batches of data. Therefore, the width of the box somewhat indicates how much the data fluctuate. The flatter the box indicates a greater concentration of data, and the shorter the endline also indicates a concentration of data, and the results show that the current state of construction of architectural heritage conservation work in Yan'an is still at a low level.

The first is the principle of objectivity. The conservation of heritage in cities involves many aspects, such as the current state of urban economic development, natural environmental factors, and urban future development planning, and the one-sidedness of the indicator orientation due to the conflict of different values should be avoided in the determination of the indicator system. The second is the principle of quantification. Architectural heritage conservation is influenced by many factors such as politics, economy, and culture, so the indicators are complex and systematic, so it is necessary to set some qualitative indicators. The final strategic principle is to be forward-looking and to formulate a long-term development plan. The RNN method is used to establish an evaluation model of environmental measures in architectural heritage conservation work, which provides a basis for the future development of architectural heritage conservation in Yan'an. The comparison of the simulation responses is shown in Figure 8, which is basically consistent with the results of the theoretical analysis and provides a sufficient analysis for the further improvement of environmental measures in architectural heritage conservation work in Yan'an in the later stage. In addition to more scientific research, best practices should be developed to open up and share knowledge about the complex interplay between environmental-like measures and historic preservation of buildings.

## 5. Conclusions

Architectural heritage conservation is a topical issue in today's society. How to conserve architectural heritage is a common concern, and the relevant results are extremely abundant. However, the evaluation and analysis of the environmental aspects of conservation has not yet received much attention. No matter what kind of documents, policies, tools, and measures are formulated, the ultimate aim is to better realize the conservation, heritage, and development of architectural heritage. The key question is whether these policies, measures, methods, and instruments have been put into practice, whether they are practical and scientific, and whether they have achieved the desired goals. In short, it is how effective the conservation is. Given that existing evaluation methods cannot provide new solutions for decision-making, the meaning of the comprehensive evaluation function is unclear, naming clarity is low, quantitative data is scarce, there are many qualitative components, and the results are not easily convincing. This paper proposes an RNN analysis method to evaluate the implementation effect of the environmental category of architectural heritage in Yan'an with greater applicability, which is basically consistent with the results of the theoretical analysis. It provides a basis for the construction of architectural heritage in Yan'an and provides a reference for the future development direction of architectural heritage in Yan'an. It is expected to draw more attention and discuss the theory of architectural heritage conservation effect evaluation together and provide a theoretical basis for realizing the conservation, inheritance, and development of architectural heritage.

## Figures and Tables

**Figure 1:** Schematic diagram of the RNN.

**Figure 2:** Actual effect evaluation framework of environmental measures in Yan'an architectural heritage protection work.

**Figure 3:** Hierarchical analysis box-line diagram.

**Figure 4:** Diagram comparing the effects of hierarchical analysis simulation.

**Figure 5:** Factor analysis method box-line diagram.

**Figure 6:** Diagram comparing the simulation effects of the factor analysis method.

**Figure 7:** RNN neural network analysis method box-line diagram.

**Figure 8:** Diagram comparing the simulation effect of RNN neural network analysis method.

## Data Availability

The dataset can be accessed upon request.

## References

[1] Lidelöw S., Örn T., Luciani A., Rizzo A. (2019). Energy-efficiency measures for heritage buildings: a literature review. *Sustainable Cities and Society*.

[2] Zan M. L., Heras V. C., Wijffels A. (2014). A value-based monitoring system to support heritage conservation planning. *Journal of Cultural Heritage Management and Sustainable Development*.

[3] Yung E. H. K., Lai L. W. C., Philip L. H. (2016). Public decision making for heritage conservation: a Hong Kong empirical study. *Habitat International*.

[4] He W. M., Wang J. (2011). Research of Yan’an Red Base area architecture from 30 years to 40 years in 20 century [C]//advanced materials research. *Trans Tech Publications Ltd*.

[5] Wu K. (2015). *Reinventing Chinese Tradition: the cultural politics of late socialism [M]*.

[6] Lin C. (2015). Red tourism: rethinking propaganda as a social space. *Communication and Critical/Cultural Studies*.

[7] Chang Q. (2019). Architectural models and their contexts in China’s 20th-century architectural heritage: an overview. *Built Heritage*.

[8] Yu C. (2016). *12 Regenerating urban waterfronts in China*.

[9] Yisan R. (2013). Conservation and proper use of historic urban heritage in China [J]. *Conservation and proper use of historic urban heritage in China*.

[10] Hao Y., Liang X., Lan Y. (2021). Numerical simulation and dynamic analysis of single-hole cliff-side loess cave dwelling under seismic actions. *Geofluids*.

[11] Revez M. J., Coghi P., Rodrigues J. D., Vaz Pinto I. (2021). Analysing the cost-effectiveness of heritage conservation interventions: a methodological proposal within project STORM. *International Journal of Architectural Heritage*.

[12] Li Y., Zhao L., Huang J., Law A. (2021). Research frameworks, methodologies, and assessment methods concerning the adaptive reuse of architectural heritage: a review. *Built Heritage*.

[13] López F. J., Lerones P. M., Llamas J., Gómez-García-Bermejo J., Zalama E. (2018). A review of heritage building information modeling (H-BIM). *Multimodal Technologies and Interaction*.

[14] Otero J. (2022). Heritage conservation future: where we stand, challenges ahead, and a paradigm shift. *Global Challenges*.

[15] Bruno S., De Fino M., Fatiguso F. (2018). Historic building information modelling: performance assessment for diagnosis-aided information modelling and management. *Automation in Construction*.

[16] Porębska A., Godyń I., Radzicki K., Nachlik E., Rizzi P. (2019). Built heritage, sustainable development, and natural hazards: flood protection and UNESCO world heritage site protection strategies in Krakow, Poland. *Sustainability*.

[17] Campiani A., Lingle A., Lercari N. (2019). Spatial analysis and heritage conservation: leveraging 3-D data and GIS for monitoring earthen architecture. *Journal of Cultural Heritage*.

[18] Gulotta D., Toniolo L. (2019). Conservation of the built heritage: pilot site approach to design a sustainable process. *Heritage*.

[19] Wang R., Liu G., Zhou J., Wang J. (2019). Identifying the critical stakeholders for the sustainable development of architectural heritage of tourism: from the perspective of China. *Sustainability*.

[20] De Medici S. (2021). Italian architectural heritage and photovoltaic systems. Matching style with sustainability. *Sustainability*.

[21] Aigwi I. E., Filippova O., Ingham J., Phipps R. (2021). From drag to brag: the role of government grants in enhancing built heritage protection efforts in New Zealand’s provincial regions. *Journal of Rural Studies*.

[22] Salameh M. M., Touqan B. A., Awad J., Salameh M. M. (2022). Heritage conservation as a bridge to sustainability assessing thermal performance and the preservation of identity through heritage conservation in the Mediterranean city of Nablus. *Ain Shams Engineering Journal*.

[23] Baranwal M., Clark R. L., Thompson J., Sun Z., Hero A. O., Venturelli O. S. (2022). Recurrent neural networks enable design of multifunctional synthetic human gut microbiome dynamics. *eLife*.

[24] Wang Y., Chen Z., Chen Z. B. (2022). Dynamic graph conv-LSTM model with dynamic positional encoding for the large-scale traveling salesman problem. *Mathematical Biosciences and Engineering*.

[25] Hu C., Martin S., Dingreville R. (2022). Accelerating phase-field predictions via recurrent neural networks learning the microstructure evolution in latent space. *Computer Methods in Applied Mechanics and Engineering*.

[26] Pannitto L., Herbelot A. (2022). Can recurrent neural networks validate usage-based theories of grammar acquisition?. *Frontiers in Psychology*.

[27] Reza S., Ferreira M. C., Machado J. J. M., Tavares J. M. R. S. (2022). A multi-head attention-based transformer model for traffic flow forecasting with a comparative analysis to recurrent neural networks. *Expert Systems with Applications*.

[28] Gou F., Wu J. (2022). Message transmission strategy based on recurrent neural network and attention mechanism in IoT system. *Journal of Circuits, Systems and Computers*.

[29] Cheng Z., Chen B., Lu R. (2022). Recurrent neural networks for snapshot compressive imaging. *IEEE Transactions on Pattern Analysis and Machine Intelligence*.

[30] Bonatti C., Mohr D. (2022). On the importance of self-consistency in recurrent neural network models representing elasto-plastic solids. *Journal of the Mechanics and Physics of Solids*.

[31] Vamosi S., Reutterer T., Platzer M. (2022). A deep recurrent neural network approach to learn sequence similarities for user-identification. *Decision Support Systems*.

[32] Meager R. (2022). Aggregating distributional treatment effects: a Bayesian hierarchical analysis of the microcredit literature. *American Economic Review*.

[33] Yao J., Guo X., Wang L., Jiang H. (2022). Understanding green consumption: a literature review based on factor analysis and bibliometric method. *Sustainability*.

[34] Pius R., Sen A. (2018). Unitarity of the box diagram. *Journal of High Energy Physics*.

